The article "Computed Tomography Texture Features and Risk Factor Analysis of Postoperative Recurrence of Patients with Advanced Gastric Cancer after Radical Treatment under Artificial Intelligence Algorithm" was published in 2022. Journal: Comput Intell Neurosci.

# Computed Tomography Texture Features and Risk Factor Analysis of Postoperative Recurrence of Patients with Advanced Gastric Cancer after Radical Treatment under Artificial Intelligence Algorithm

**DOI:** 10.1155/2022/1852718

**Published:** 2022-05-24

**Authors:** Zhiwu Zhou, Mei Zhang, Chuanwen Liao, Hong Zhang, Qing Yang, Yu Yang

**Affiliations:** ^1^Department of Gastrointestinal Surgery, Jiangxi Provincial People's Hospital, Nanchang 330006, Jiangxi, China; ^2^Department of Medical Imaging, Jiangxi Provincial People's Hospital, Nanchang 330006, Jiangxi, China; ^3^Department of Neurosurgery, Jiangxi Provincial People's Hospital, Nanchang 330006, Jiangxi, China

## Abstract

Computer tomography texture analysis (CTTA) based on the V-Net convolutional neural network (CNN) algorithm was used to analyze the recurrence of advanced gastric cancer after radical treatment. Meanwhile, the clinical characteristics of patients were analyzed to explore the recurrence factors. 86 patients who underwent the advanced radical gastrectomy for gastric cancer were retrospectively selected as the research objects. Patients were divided into the no-recurrence group (30 cases) and the recurrence group (56 cases) according to whether there was recurrence after radical treatment. CTTA was performed before and after surgery in both groups to analyze the risk factors for recurrence. The results showed that the dice coefficient (0.9209) and the intersection over union (IOU) value (0.8392) of the V–CNN segmentation effect were signally higher than those of CNN, V-Net, and context encoder network (CE-Net) (*P* < 0.05). The mean value of arterial phase and portal phase (65.29 ± 9.23)/(79.89 ± 10.83), kurtosis (3.22)/(3.13), entropy (9.99 ± 0.53)/(9.97 ± 0.83), and correlation (4.12 × 10^−5^/4.21 × 10^−5^) of the recurrence group was higher than the no-recurrence group, while the skewness (0.01)/(−0.06) of the recurrence group was lower than that of the no-recurrence group (*P* < 0.05). Patients aged 60 years old and above, with a tumor diameter of 6 cm and above, and in the stage III/IV in the recurrence group were higher than those in the no-recurrence group, and patients with chemotherapy were lower (*P* < 0.05). To sum up, age, tumor diameter, whether chemotherapy should be performed, and tumor staging were all the risk factors of postoperative recurrence among patients with gastric cancer. Besides, CT texture parameter could be used to predict and analyze the postoperative recurrence of gastric cancer with good clinical application values.

## 1. Introduction

As one of the most common malignant tumors in the world, gastric cancer not only has a high incidence that ranks fourth among malignant tumors but also has a high fatality rate that is the second-highest [1]. Hence, the treatment of gastric cancer has always been the focus of clinical research, especially in China. With the continuous development of clinical diagnosis and treatment technology, the diagnosis and treatment of gastric cancer have made certain progress. At present, the ubiquitous clinical treatment for gastric cancer is surgical treatment, and radical gastrectomy is the most common surgical treatment [2], combined with chemotherapy and radiotherapy [3]. Radical gastrectomy-combined chemotherapy and radiotherapy can improve the therapeutic effect of patients with gastric cancer to a certain extent, but there are still poor prognoses, and even postoperative recurrence and/or metastasis [4]. Consequently, the characteristics and risk factors of postoperative recurrence of gastric cancer deserve attention. Reasonable and accurate analysis of risk factors has certain significance to reduce the probability of recurrence after radical gastrectomy [5]. Although there are some relevant explorations on postoperative recurrence and metastasis of gastric cancer in recent years, there are still few on the relationship among the possibility of recurrence, modes, and clinical and pathological factors.

The article "Computed Tomography Texture Features and Risk Factor Analysis of Postoperative Recurrence of Patients with Advanced Gastric Cancer after Radical Treatment under Artificial Intelligence Algorithm" was published in 2022. Journal: Comput Intell Neurosci.

Histopathological features are the crucial factors that affect the prognosis of patients with gastric cancer [6]. The gastroscopic biopsy is an invasive procedure that cannot be adopted for postoperative review [7]. Computer tomography (CT) has been widely recognized in the examination of clinical diseases due to its noninvasive methods, affordable price, and simple operation, especially the multidetector CT (MDCT). However, the imaging scanning technique is only anatomic, and its diagnostic scope is limited. Then, CT texture analysis (CTTA) has been proposed and widely used in the differentiation, classification, and prognosis of benign and malignant tumors [8]. According to some investigations, texture parameters can be used to differentiate the degree of gastric cancer and evaluate the prognosis of patients [9, 10]. CTTA refers to the evaluation of tumor heterogeneity by using pixel distribution and relationships in CT images. The main process includes image acquisition, lesion segmentation, feature extraction, feature analysis, and model establishment [11]. To improve the accuracy of CTTA, artificial intelligence (AI) algorithm will be combined to improve the above steps to improve the image segmentation effect. The convolutional neural network (CNN) algorithm is a common algorithm used in medical images [12]. Nevertheless, the simple CNN algorithm is not often precise enough in image segmentation. Therefore, a V-Net-CNN (V–CNN) algorithm is proposed [13], which improves the CNN by optimizing the loss function of the V-Net's structure to improve the inaccuracy of segmentation. Besides, the improved V–CNN algorithm has high accuracy in segmentation for CT images.

The article "Computed Tomography Texture Features and Risk Factor Analysis of Postoperative Recurrence of Patients with Advanced Gastric Cancer after Radical Treatment under Artificial Intelligence Algorithm" was published in 2022. Journal: Comput Intell Neurosci.

Hence, V–CNN algorithm-based CT texture analysis was adopted to analyze the patients with postoperative recurrence after progressive gastric cancer radical surgery to further investigate the clinical application values of CT texture analysis in postoperative recurrence after the surgery of gastric cancer and the factors causing postoperative recurrence. The differences between the patients with recurrent gastric cancer and without recurrent gastric cancer were compared. Besides, the clinical characteristics of patients were analyzed to investigate the factors resulting in recurrence, which provided the reasonable and effective research basis for the improvement of the diagnostics and therapeutic effects on recurrent gastric cancer and the postoperative prognosis of patients.

## 2. Methods

### 2.1. The Research Objects

Eighty-six patients who underwent the advanced radical gastrectomy for gastric cancer in hospital from January 2018 to December 2020 were retrospectively selected as the research objects. Complete clinical data and follow-up data were collected. There were 62 male patients and 24 female patients, ranging in age from 30 to 80 years old, with an average age of (56.32 ± 12.89) years old. There were 30 patients whose tumors occurred at the junction of the esophagus and stomach, 48 patients whose tumors occurred in the distal stomach, and 8 patients whose tumors occurred in the whole stomach. There were 58 cases with high/medium differentiation and 28 cases with low/undifferentiated differentiation. There were 29 patients in stage I/II of the tumor, node, and metastasis (TNM) and 57 patients in stage III/IV of TNM. The patients were divided into the no-recurrence group (30 cases) and the recurrence group (56 cases) according to whether the patients had recurrence after surgery. CTTA was performed before and after surgery for patients in the two groups, the CT texture characteristics of patients after recurrence were summarized, and the risk factors that affected the recurrence were analyzed. This study had been approved by the ethics committee of hospital, and all subjects included had signed the informed consent forms.

The inclusion criteria were as follows: I. the pathological stage of all patients was based on the American Joint Committee on Cancer (AJCC) gastric cancer stage (8th edition) [14]; II. all patients underwent the CT examination before and after surgery; III. patients with complete clinical data; IV. patients and their family members signed the informed consent; and V. patients with complete follow-up data for 2 years or more.

The article "Computed Tomography Texture Features and Risk Factor Analysis of Postoperative Recurrence of Patients with Advanced Gastric Cancer after Radical Treatment under Artificial Intelligence Algorithm" was published in 2022. Journal: Comput Intell Neurosci.

The exclusion criteria were as follows: I. patients with other serious organ dysfunction and infectious diseases; II. patients with intermediate or advanced cancer stages; III. patients with missing CT images; and IV. patients who received antitumor therapy before the surgery.

### 2.2. CT Image Segmentation Algorithm

CT of the stomach is usually obtained by scanning layer by layer. However, the gastric wall is usually located in the upper abdomen, and the gastric wall is irregular. Hence, data enhancement is not suitable for the processing of gastric CT images. The new image was obtained by adding random noise to simulate a reasonable CT image for supplementing the image parameters. To retain the original features of the image, linear random perturbation was inserted to keep the variation range of CT pixels within a certain range. (1) showed the specific expression.

(1) $$\begin{array}{c} Q^{*}=Q+\cos\left(180+\alpha^{1}\right)\cdot {\left(-2\times \;\log\;\alpha^{2}\right)}^{1/2}. \end{array}$$

In (1), *Q*^*∗*^ is the inserted pixel value, *Q* represented the current pixel value, and *α*^1^ and *α*^2^ represented the random floating-point numbers. After the processed CT image was obtained, it was necessary to collect the image features. The traditional CNN algorithm led to the loss of vital image information in the process of image feature extraction. Consequently, the adopted feature map was multiplied by a certain weight value, and (2) showed the specific weight calculation.

(2) $$\begin{array}{c} W^{i}=\frac{\left|GAP\left(F^{i}\right)\right|}{\sum_{i=1}^{4}\left|GAP\left(F^{i}\right)\right|}. \end{array}$$

In (2), *i* expressed the number of convolutional layers, *W*_*i*_ expressed the weight value, *GAP* expressed the global average pooling (GAP), and *F*_*i*_ expressed the convolutional output of the *i*-th layer.

Cross-entropy [15] (CE)/dice coefficient loss function (dice loss) was used in the traditional image segmentation. The adoption of loss function was relatively pervasive, but the effect of the loss function in gastric wall segmentation was not ideal. Then, the level set loss function (L S loss) was proposed [16]. The function expressions of the L S loss method in the deep learning network were shown as

(3) $$\begin{array}{c} F_{L\left(\phi \right)}=\mu \times \text{length}\left(\phi \right). \end{array}$$

(4) $$\begin{array}{c} F_{A\left(\phi \right)}=\chi \times \text{Area}\left(\phi \right). \end{array}$$

(5) $$\begin{array}{c} F_{c_{1}\left(\phi \right)}=\delta_{1}\sum_{\Pi }{\left|\mu_{0}\left(x,y\right)-c_{1}\right|}^{2}H\left(\phi \left(x,y\right)\right)\text{d}x\text{d}y. \end{array}$$

(6) $$\begin{array}{c} F_{c_{2}\left(\phi \right)}=\delta_{2}\sum_{\Pi }{\left|\mu_{0}\left(x,y\right)-c_{2}\right|}^{2}\left(1-H\left(\phi \left(x,y\right)\right)\right)\text{d}x\text{d}y. \end{array}$$

(7) $$\begin{array}{c} F_{\left(c_{1},c_{2}\left(\phi \right)\right)}=F_{L\left(\phi \right)}+F_{A\left(\phi \right)}+F_{c_{1}\left(\phi \right)}+F_{c_{2}\left(\phi \right)}. \end{array}$$

In equations (3)–(7), *μ*, *χ*, *δ*_1_, and *δ*_2_ all represented the quantitative parameters, which were all greater than 0. *ϕ* represented the level set function, *c*_1_ represented the average pixel value inside the curve, and *c*_2_ represented the average pixel value outside the curve. length(*ϕ*) represented the regularization term of curve length, Area(*ϕ*) represented the regularization term of curve area, *μ*_0_ represented pixel value, (*x*, *y*) represented image position, Π represented the whole image area, and *H* represented the step function (differentiable). (8) showed the specific expression.

(8) $$\begin{array}{c} H\left(x\right)=\frac{1}{180\cdot }arc\cdot \;\tan\left(\varepsilon x+60\right). \end{array}$$

In (8), *ε* expressed the hyperparameter, and its main function was raising the gradient of the function. However, the L S loss function could be adopted for the segmentation of single edge objects, and the segmentation effect of the inner and outer edges of the gastric wall was insufficient. In equations (9)–(12), it was defined as the regularization level set loss function (LSR loss) to constrain the internal detail features of the gastric wall.

(9) $$\begin{array}{c} F_{c_{l1}\left(\phi \right)}=\frac{1}{\delta_{1}}\sum_{\Pi }{\left|G_{l}\left(x,y\right)-c_{l1}\right|}^{2}H\left(\phi \left(x,y\right)\right). \end{array}$$

(10) $$\begin{array}{c} F_{c_{l2}\left(\phi \right)}=\frac{1}{\delta_{2}}\sum_{\Pi }{\left|G_{l}\left(x,y\right)-c_{l2}\right|}^{2}\left(1-H\left(\phi \left(x,y\right)\right)\right). \end{array}$$

(11) $$\begin{array}{c} F_{c_{l3}\left(\phi \right)}=\frac{1}{\delta_{3}}\sum_{\Pi }{\left|G_{l}\left(x,y\right)-\phi \left(x,y\right)\right|}^{2}. \end{array}$$

(12) $$\begin{array}{c} LSR\text{ loss}=F_{c_{l1}\left(\phi \right)}+F_{c_{l2}\left(\phi \right)}+F_{c_{l3}\left(\phi \right)}. \end{array}$$

In equations (9)–(12), *G*_*l*_(*x*, *y*) represented the pixel value of ground truth and *ϕ*(*x*, *y*) represented the predicted pixel value.

(13) $$\begin{array}{c} c_{l1}\left(\phi \right)=\frac{\sum_{\Pi }G_{l}•H\left(\phi \left(x,y\right)\right)}{\sum_{\Pi }H\left(\phi \left(x,y\right)\right)},\\ c_{l2}\left(\phi \right)=\frac{\sum_{\Pi }G_{l}•\left(1-H\left(\phi \left(x,y\right)\right)\right.}{\sum_{\Pi }\left(1-H\left(\phi \left(x,y\right)\right)\right.}. \end{array}$$

LSR loss had the characteristics of traditional-level set function edge optimization and could suppress the over-fitting phenomenon. To evaluate the segmentation effect of the algorithm, the dice coefficient and intersection over union (IOU) were used for evaluation. (14) and (15) showed the calculation methods.

(14) $$\begin{array}{c} IOU=\frac{\left|M^{G}⊙M^{P}\right|}{\left|M^{G}\right|⊗\left|M^{P}\right|}. \end{array}$$

(15) $$\begin{array}{c} \text{Dice}=\frac{2\left|M^{G}⊙M^{P}\right|}{\left|M^{G}\right|⊕\left|M^{P}\right|}. \end{array}$$

In (14) and (15), *M*^*G*^ expressed the ground truth and *M*^*P*^ expressed the predicted value outputted by the neural network. The dice coefficient and IOU values ranged from 0 to 1. The higher the result was, the higher the segmentation accuracy was.

The article "Computed Tomography Texture Features and Risk Factor Analysis of Postoperative Recurrence of Patients with Advanced Gastric Cancer after Radical Treatment under Artificial Intelligence Algorithm" was published in 2022. Journal: Comput Intell Neurosci.

### 2.3. Methods of Examination

All patients received the examinations by the same surgeon with the same instrument, namely, the 64-slice multi-slice spiral CT. Before the examination, patients were asked to fast for 6 hours, and they were placed in the supine position during the examination. The scan area was from the diaphragmatic apex to the anterior superior iliac spine. The scanning parameters were as follows. The tube voltage was 120 kV, tube current was 200–260 mA, the thickness was 5 mm, layer spacing was 5 mm, the field of view was 35–50 cm, the matrix was 512 × 512, and the time was 0.7 s. Then, the contrast agent was injected. After 30 seconds, the images of arterial phase were obtained. After 70 seconds, the images of portal vein phase were obtained. After that, the obtained images were imported in the format of digital imaging and communications in medicine (DICOM).

### 2.4. The Follow-Up Visit

The follow-up visit was performed for more than two years through the outpatient review results, telephone consultation, and inpatient medical records. During the follow-up period, the serum carcinoembryonic antigen, carbohydrate antigen 19–9 (CA19-9), abdominal CT, ultrasound, and other comprehensive examinations were performed to examine whether the patients had recurrence or metastasis after the surgery.

### 2.5. Observation Indexes

The processed CT images were imported into the CT kinetics for the texture parameter measurement and analysis. The delineation of the region of interest (ROI) was performed by an experienced physician. The corresponding gray histogram and a series of texture parameters based on gray-level co-occurrence matrix (GLCM) were automatically generated by this software. Subsequently, mean value, skewness, kurtosis, entropy, and correlation were extracted for comparison and analysis.

The article "Computed Tomography Texture Features and Risk Factor Analysis of Postoperative Recurrence of Patients with Advanced Gastric Cancer after Radical Treatment under Artificial Intelligence Algorithm" was published in 2022. Journal: Comput Intell Neurosci.

The differences between the general data and clinical case data of the two groups were compared. Factors that caused the postoperative recurrence were analyzed, including univariate and multivariate analyses.

### 2.6. Statistical Methods

SPSS 22.0 was employed for data statistics and analysis. The statistic of the quantity was expressed by *x* ± *s*. The *t*-test was adopted. Percentage (%) was how data statistics were expressed. Logistic analysis was used to analyze the risk factors of postoperative recurrence, and the difference was statistically significant by using the *χ*^2^ test. The difference was statistically significant with *P* < 0.05.

## 3. Results

### 3.1. Comparison of Segmentation Effects

The V–CNN structure was compared with CNN, V-Net, and CE-Net structures through dice coefficient and IOU values. The dice coefficient of V–CNN, CNN, V-Net, and CE-Net was 0.9209, 0.8442, 0.8522, and 0.8632, respectively. IOU values of V–CNN, CNN, V-Net, and CE-Net were 0.8392, 0.7671, 0.7272, and 0.7727, respectively. According to the comparison, the dice coefficient and IOU values of the V–CNN segmentation effect were remarkably higher than those of CNN, V-Net, and CE-Net (*P* < 0.05) (Figure 1).  Figure 2 shows the specific diagrams of segmentation effects. The segmentation contour of the algorithm in this experiment was consistent with the original image.

### 3.2. The Results of CT Texture Analysis

Mean value, skewness, kurtosis, entropy, and correlation of patients in the arterial phase and portal phase were compared between the two groups. In the arterial stage, the mean value (65.29 ± 9.23), kurtosis (3.22), entropy (9.99 ± 0.53), and correlation (4.12 × 10^−5^) in the recurrence group were higher than those in the no-recurrence group, and the skewness (0.01) was lower than that in the no-recurrence group (*P* < 0.05) (Figure 3). In the portal vein stage, the mean value (79.89 ± 10.83), kurtosis (3.13), entropy (9.97 ± 0.83), and correlation (4.21 × 10^−5^) in the recurrence group were higher than those in the no-recurrence group, and the skewness (−0.06) was lower than that in the no-recurrence group (*P* < 0.05).

### 3.3. Clinical Data Statistics and Risk Factor Analysis

The general clinical data and pathological conditions of 56 patients in the recurrence group and 30 patients in the no-recurrence group were statistically analyzed.

#### 3.3.1. Case Data Statistics

In terms of gender distribution, there were 40 male patients (71.43%) and 16 female patients (28.57%) in the recurrence group. There were 22 male patients (73.33%) and 8 female patients (26.67%) in the no-recurrence group. In terms of age distribution, 21.43% (12/56) of patients were under 60 years old, and 78.57% (44/56) were 60 years old and above in the recurrence group. In the no-recurrence group, 76.67% (23/30) of patients were under 60 years old, and 23.33% (7/30) were 60 years old and above, as shown in Figure 4.

The article "Computed Tomography Texture Features and Risk Factor Analysis of Postoperative Recurrence of Patients with Advanced Gastric Cancer after Radical Treatment under Artificial Intelligence Algorithm" was published in 2022. Journal: Comput Intell Neurosci.

#### 3.3.2. Comparison of Tumor and Treatment Information

In terms of preoperative tumor diameter, there were 6 patients (10.71%) with tumor diameter below 6 cm in the recurrence group and 50 patients (89.28%) with tumor diameter above 6 cm. In the no-recurrence group, 27 patients (90%) had tumors with a diameter below 6 cm, while 3 patients (10%) with tumor diameter above 6 cm. In terms of TNM stage, the proportion of patients with stage I/II and stage III/IV was 16.07% (9/56) and 83.93% (47/56) in the recurrence group. In the no-recurrence group, the proportion of stage I/II patients was 86.67% (26/30), and that of stage III/IV patients was 13.33% (4/30). In the recurrence group, 20 cases (35.71%) had tumors located at the junction of esophagus and stomach, 31 cases (55.36%) at the distal stomach, and 5 cases (8.93%) at the whole stomach. In the no-recurrence group, there were 10 cases (33.33%) at the junction of esophagus and stomach, 17 cases (56.67%) at the distal stomach, and 3 cases (10%) at the whole stomach. In terms of whether patients received chemotherapy, only 7 patients (12.5%) received chemotherapy in the recurrence group and 49 patients (87.5%) did not. In the no-recurrence group, 13 patients (43.33%) received chemotherapy, while 17 patients (56.67%) did not (Figures 5 and 6).

#### 3.3.3. Risk Factor Analysis

According to the above statistical results, there were insignificant statistical differences in the proportion of male and female patients and the location distribution of tumor occurrence between the two groups (*P* > 0.05). The proportion of patients aged 60 years and above, with a tumor diameter of 6 cm and above, and in tumor stage III/IV in the recurrence group was greatly higher than that in the no-recurrence group, and the proportion of patients who underwent chemotherapy was lower than that in the no-recurrence group (*P* < 0.05). Univariate analysis was performed only for the recurrence group, and the results were consistent with the above conclusions. Patients' age, TNM stage, tumor diameter, and chemotherapy or not were associated with postoperative recurrence.  Table 1 shows the multi-factor analysis results, which indicated that age, tumor diameter, chemotherapy, and TNM stage were the main factors that affected postoperative recurrence of laparoscopic radical gastrectomy for gastric cancer (*P* < 0.05).

The article "Computed Tomography Texture Features and Risk Factor Analysis of Postoperative Recurrence of Patients with Advanced Gastric Cancer after Radical Treatment under Artificial Intelligence Algorithm" was published in 2022. Journal: Comput Intell Neurosci.

## 4. Discussion

Attention needs to be paid to both the early and late stages of gastric cancer. The atypical manifestations of early gastric cancer can easily lead to the late development of treatment. Therefore, the examination of early gastric cancer and the effective treatment of late gastric cancer is the focus of clinical research [17]. Moreover, postoperative recurrence of patients with gastric cancer has also been the focus of clinical attention, including examination, diagnosis, and analysis of risk factors that affect postoperative recurrence.

CT images were used for texture analysis to understand the difference of CT texture parameters between recurrent and nonrecurrent patients. Since CTTA requires feature segmentation and extraction of lesions, the V–CNN algorithm is adopted for the processing of CT images to improve the accuracy of image segmentation. V–CNN was improving the image segmentation effect by optimizing loss function, and the V–CNN algorithm was improved by LSR loss. The evaluation results reflected that the dice coefficient (0.9209) and IOU value (0.8392) of the V–CNN segmentation effect were markedly higher than those of CNN, V-Net, and CE-Net (*P* < 0.05). The improvement of the V-Net network by LSR loss was helpful to improve the segmentation effect of the CNN algorithm. Furthermore, the accuracy of the V-Net and the original segmentation algorithm improved by LSR loss was increased by 6%, which provided support for the results of this experiment [18]. Aghababaie et al. (2020) [19] also used the V-Net based on the CNN algorithm to segment the images of stomach examination, and the results suggested that this method could be transformed into emerging clinical skills. Besides, Xu et al. (2020) [20] used the improved V-Net for the automatic segmentation of maxillary sinus CT images, and the adoption effect was good.

Under the premise of the effective segmentation algorithms, the texture parameters of gastric CT of two groups were compared. In the arterial phase and portal phase, the mean value (65.29 ± 9.23)/(79.89 ± 10.83), kurtosis (3.22)/(3.13), entropy (9.99 ± 0.53)/(9.97 ± 0.83), and correlation (4.12 × 10^−5^/4.21 × 10^−5^) in the recurrence group were higher than those in the no-recurrence group, while the skewness (0.01)/(−0.06) was lower than that of the no-recurrence group (*P* < 0.05). Masci et al. (2022) [21] proposed that CTTA could be used for the prediction and diagnosis of gastric cancer. Liu et al. (2018) [22] proposed that CTTA was correlated with the TNM stage of gastric cancer to a certain extent. The higher the mean, kurtosis, entropy, and correlation were, the lower the skewness was, and the higher the TNM was. Zeydanli and Kilic (2021) [23], and Liu et al. (2017) [24] proposed that CTTA was conducive to the classification of gastric neoplasm and prediction of gastric adenocarcinoma differentiation. CT images of patients without recurrence were compared with those of patients with recurrence. Hence, patients in the no-recurrence group had no TNM stage. The TNM stage of the no-recurrence group was lower than that of the recurrence group, which was consistent with the research results. Meanwhile, there were no significant differences in gender and distribution of tumor location between the two groups (*P* > 0.05). Patients aged 60 years and older, with a tumor diameter of 6 cm and above, and in stage III/IV in the recurrence group were higher than those in the no-recurrence group, and patients who received chemotherapy were lower than those in the no-recurrence group (*P* < 0.05). Therefore, postoperative recurrence was correlated with age, TNM stage, tumor diameter, and chemotherapy or not, but not with gender or disease location. According to the results of multi-factor analysis, age, tumor diameter, chemotherapy or not, and TNM stage were the main factors that affected the postoperative recurrence of laparoscopic radical gastrectomy for gastric cancer (*P* < 0.05). Zou et al. (2021) [25], Chen et al. (2021) [26], Nakagawa et al. (2018) [27], and Jin et al. (2020) [28] proposed that tumor stage, tumor size, patients' age, and postoperative treatment affected the recurrence of gastric cancer, which supported the results of this experiment. Moreover, inflammatory factors and venous infiltration can also affect the surgical prognosis and recurrence of patients with gastric cancer [29, 30], which was not involved in this experiment. Hence, it will be further explored in the future.

The article "Computed Tomography Texture Features and Risk Factor Analysis of Postoperative Recurrence of Patients with Advanced Gastric Cancer after Radical Treatment under Artificial Intelligence Algorithm" was published in 2022. Journal: Comput Intell Neurosci.

## 5. Conclusion

To conclude, age, tumor diameter, whether chemotherapy should be performed, and tumor staging were all the risk factors of postoperative recurrence among patients with gastric cancer, which needed to be focused on. In addition, CT texture parameter could be used to predict and analyze the postoperative recurrence of gastric cancer with good clinical application values. Nonetheless, through the literature search, more factors affected postoperative recurrence than the mentioned above, and this experiment is not comprehensive enough. Further investigation and analysis are needed. Furthermore, CTTA technology has a good adoption prospect in clinical research and analysis of gastric cancer diseases. Besides, the research results demonstrated that CTTA technology showed a good development prospect in the clinical research and analysis of gastric cancer disease and was worthy of clinical promotion.

## Figures and Tables

**Figure 1:** Comparison of the evaluation results of segmentation effects. ^∗^Comparison with V–CNN algorithm, *P* < 0.05.

**Figure 2:** Diagrams of segmentation effects. If the first line was set to be the first layer of the slice image, the first, second, and fourth gastric CT slice images were from top to bottom.

**Figure 3:** CT texture analysis results and recurrence CT images. ^*∗*^Comparison with recurrence group, *P* < 0.05.

**Figure 4:** Comparison of general data. ^*∗*^Comparison with recurrence group, *P* < 0.05.

**Figure 5:** Comparison of examination results.

**Figure 6:** Comparison of treatment methods. ^*∗*^Comparison with recurrence group,*P* < 0.05.

**Table 1:** Multivariate analysis of postoperative recurrence.

Factors	Age	TNM stage	Tumor diameter	Chemotherapy or not
Regression coefficient	1.012	9.987	1.031	−0.891
Word	6.331	5.561	6.877	7.261
Relative risk	0.987	1.309	1.209	1.342
*P*	0.012^*∗*^	0.021^*∗*^	0.014^*∗*^	0.019^*∗*^
95% CI	[1.023, 1.536]	[1.022, 1.655]	[1.082, 1.321]	[0.921, 1.621]

*Note.* ^*∗*^Comparison suggested statistical difference, *P* < 0.05.

## Data Availability

The data used to support the findings of this study are available from the corresponding author upon request.
